RETRACTED

# Sexual reproductive health service utilization and associated factors among undergraduate students of Addis Ababa University in Ethiopia

**DOI:** 10.1186/s41043-023-00363-9

**Published:** 2023-03-17

**Authors:** Bethel Mekbib, Dereje Bayissa Demissei

**Affiliations:** 1 Department of Reproductive Health, Sante Medical College, Addis Ababa, Ethiopia; 2 St. Paul’s Hospital Millennium Medical College, Addis Ababa, Ethiopia

**Keywords:** Sexual reproductive health service utilization, SRH service

## Abstract

**Background:**

Making clinical services attractive to the younger generation has remained a challenge. Students in higher education continue to underutilize sexual and reproductive health services. This group is exposed to a very hostile environment and has a highly mobile and unprotected lifestyle, often resulting in an early sexual debut, physical and drug abuse, and sexually transmitted infections.

**Objective:**

The aim of this study was to assess sexual reproductive health services and associated factors among undergraduate students of Addis Ababa University 2022.

**Method:**

An Institution-based cross-sectional study was been conducted among 419 randomly selected students and data were collected by using semi-structured and pre-tested questionnaire. Data were entered to Epi info data 7.0 and exported to SPSS version 21.0 for further analysis. Both binary and multiple logistic regression analysis was used to identify factors at *P* < 0.05 with 95% CI and AOR.

**Results:**

When queried, all 419 youths agreed to participate in the study, for a response rate of 100%. The mean age of the respondents was 22 years. The majority of respondents (371, 88.5%) were between the ages of 19 and 24, and 221 (52.7%) were female. More than half of those polled (273, or 65.2%) were third-year students, while 59, or 14.1%, were first-year students. About 206 (49.2%) of participants lived with their father and mother, but 138 (32.9%) had never discussed sexual and reproductive health. Finally, 205 respondents (or 48.9%) had ever used the Sexual and Reproductive Health Services. College of business (AOR (95% CI) 3.546 (1.62–7.79), respondents who live with only their mother (AOR (95% CI) 9.37 (2.78–31.51) and who live alone (AOR (95% CI) 5.75 (2.40–13.79), positive attitude toward SRHS (AOR (95% CI) 3.15 (1.71–5.80), good knowledge (AOR (95% CI) 4.16 (2.27–7.64), frequency of discussing SRHS(AOR (95% CI) 1.93 (1.12–3.346), Convenient location of youth RHs (AOR (95% CI) 8.31 (1.61–42.93), Fee of RH services (AOR (95% CI) 12.34 (6.48–23.49) and Satisfied to received RH services (AOR (95% CI) 4.59 (2.54–8.33) were independent predictors of utilized SRHS among undergraduate students.

RETRACTED

**Conclusion and recommendation:**

The prevalence of utilization of sexual and reproductive health services was determined to be low in this study, with identified factors increasing the likelihood of utilization being attitude, knowledge, satisfaction, discussion, fee for RH services, and location, in that order. On the other hand, poor knowledge and a negative attitude toward SRHS posed risks that contributed to reproductive health issues, so we worked on advocating for services that were available in a nearby location and raising awareness. Therefore, policymakers and health planners would be better off strengthening the urgent need to ensure adequate SRHS, knowledge, and attitude building among undergraduate students in higher education in Ethiopia.

## Introduction

Reproductive health is essential for a responsible, satisfying, healthy reproductive system and a safer sexual life. Adolescents' reproductive health is becoming increasingly important, as 1.7 million people lose their lives prematurely due to reproductive health problems. It is critical during adolescence and adulthood and affects the health of the next generation [1]. Due to these reasons, adolescent’s reproductive health (RH) is becoming ever more important component of global health. Significant physiological, psychological, and social changes occur during adolescence. More than one-third of the Ethiopian population is aged between 15 and 24 and is most vulnerable to a range of sexual and reproductive health problems. Many youths are less informed about reproductive health services and less comfortable accessing those services than adults [2–4].

Youths are less informed about reproductive health services, less experienced, and less comfortable accessing health services for reproductive issues than adults. Focusing on adolescent reproductive health is both a challenge and an opportunity for health care providers. Adolescence is generally a healthy period of life, but many youths are less informed about reproductive health services [5, 6].

Limited access and low utilization of reproductive health care and services for young people contribute to and exacerbate many of the RH problems. These problems could be early childbearing, an early sexual debut, or sexually transmitted infections (STIs) including HIV/AIDS. Over a quarter of all pregnant youth and adolescents feel that their pregnancies are mistimed, reflecting this population's limited access to family planning (FP) and other RH services. Efforts have been made to address different reproductive health problems at different levels, including scaling-up and institutionalizing youth-friendly services (YFS) through intensive capacity building [5–8]. Ethiopia has been supporting efforts to increase access to sexual and reproductive health services for young people. This includes the scaling-up and institutionalization of youth-friendly services (YFS) through intensive capacity building at all levels of the health system [9, 10].

RETRACTED

However, the effects of all these efforts have not been well understood across the Ethiopian high schools and preparatory schools as is evidenced by persistent reproductive health problems and challenges to the youth [11, 12]. Young people are at high risk for reproductive health problems due to poor communication, cultural norms, poor service utilization, and low availability and accessibility of health institutions and health care providers. Reasons for low reproductive health service (RHS) utilization may include feelings of discomfort, fear of being seen by parents and others, and embarrassment while seeking reproductive health care. The precise reasons for the alleged low utilization of RH services are unknown. Utilization of sexual and reproductive health care is a major public health problem in developing countries most specifically among youths; this study is therefore significant to investigate the magnitude and associated factors among undergraduate students of Addis Ababa University. This study aimed to assess service utilization on reproductive health, service preference, and associated factors among undergraduate students in Addis Ababa University.

## Methods

### Study setting

An institutional-based cross-sectional design was conducted among undergrad students of Addis Ababa University at a selected college from July to April 2022. Addis Ababa is the capital of Ethiopia and is located in the central part of the country. Addis Ababa University (AAU) is the oldest and largest higher education and research institution in Ethiopia and has been a leading center for teaching, learning, research, and community services. The study was conducted in Addis Ababa, the capital city of the Federal Democratic Republic of Ethiopia, with a population of 2,646,000. Females outnumber males (51.9% and 48.1%, respectively), and the city is one of the most densely populated towns with a population density of 4991.1 per square kilometer. Addis Ababa University has 47,610 students (29,872 undergraduate, 15,398 masters, and 2340 PhD students) and 8709 staff (3110 academics, 4346 administrative support staff, and 1253 health professionals). It runs 70 undergraduate and 293 graduate programs (72 PhD and 221 Masters) and various specializations in health sciences. In recent years, the university has been undertaking reform schemes to cope with and respond to the fast-changing national and international educational dynamics. It has 10 colleges, 4 institutes that run both teaching and research, and 6 research institutes that predominantly conduct research. Within these academic units, there are 55 departments, 12 centers, 12 schools, and 2 teaching hospitals.

RETRACTED

### Sample size determination and sampling procedure

The sample size was determined using the single population proportion formula (54.6%). Students were stratified on two faculties, namely health science and non-health science faculties, assuming that there is a difference in knowledge on sexual and reproductive health matters between the two groups since there is no particular outcome that will be within the 5% margin of error and 95% confidence interval of certainty (alpha = 0.05) [13]. The final total sample size calculated was 419 from the single population formula. The calculated sample size of 419 was proportionally allocated to three colleges based on the number of students selected by lottery. Then a systematic sampling technique was applied to select the participants from each institution. For each selected health institution, the sampling interval (Kth) is calculated by dividing 2110 by 419, which equals 5. Then, to select the first client from the sampling interval, simple random sampling (the lottery method) was used. As a result, 57 came from the law college, 186 from the business college, and 177 from the EIABC college. The sampled client who utilized the RHS services and all undergraduate students of Addis Ababa University who agreed to participate in the study during the study period were interviewed.

### Data collection tool and procedure

A pre-tested, self-administered, structured questionnaire in the English version was adopted from a study conducted, and all the variables of interest were assessed accordingly. Adama University, a university near Addis Abeba, was the pre-test questioner. For qualitative data, by using the interview guide tool for in-depth interviews, information will be generated from key informants like youth club members, AIDS club members, and gender focal persons, as well as student clinic health care providers. Voice recorders and field notes are used to capture the information.

### Data entry and analysis

This study produced both quantitative and qualitative data. Quantitative data were analyzed through the Statistical Package for Social Scientists (SPSS) for Windows version 21.0, a data entry program. Editing was done to ensure the data was correct, accurate, and consistent. Numbers were used to code the data and put it into categories for easy analysis. Bivariate and multivariate analyses were due to factors influencing various SRH aspects. Both binary and multivariable analyses were due to factors influencing various SRH aspects. Multivariable analysis was done using logistic regression to establish any effect of independent and dependent variables while controlling for confounders. The qualitative data were analyzed using a content approach. The emerging themes were the understanding of sexual and reproductive health, the various SRH challenges and where they seek help, their thoughts on the use of SRH services, and what should be done to improve their SRH. Findings were presented in the form of charts, graphs, and frequency distribution tables to facilitate the description and explanation of the study findings.

RETRACTED

## Operational definition of term

*Health system-related question* It is related with time, cost, and person.

*Knowledge and practice of service* If the respondents mentioned at least half on their own, they were considered to have good knowledge; otherwise, they were considered to have poor.

*RH health* A state of complete physical, emotional, mental and social well-being concerning sexuality; not merely the absence of disease, dysfunction or infirmity.

*Youth-friendly reproductive health service* Services that are accessible, acceptable and appropriate for the youth. They are in the right place at the right price and delivered in the right style to be acceptable to young people and are effective, safe and affordable. They include counselling, family planning, voluntary counselling and testing and treatment of sexually transmitted infections.

*Attitude of youth toward RH service* If the respondents mentioned at least half on their own, they were considered to have good knowledge; they were considered to have good attitude whereas those respondents who scored below the mean score were categorized as negative attitudes toward RHS.

*Access* It is the extent to which a person can obtain appropriate services at a cost and effort that is both acceptable to them personally and within the means of a large majority in a given population.

*Cost affordability* when the clients respond the payment for RH services are affordable.

*Serious problem* It denotes students who are not feeling well (sick) at the time of data collection.

## Results

### Socio-demographic characteristics

When queried, all 419 youths agreed to participate in the study for a response rate of 100%. Fifty-two percent of the respondents were female 221 (52.7), and the mean age of respondent was 22 years. With majority of respondents, 371 (88.5%) were in the age group of 19–24 followed were 24 and more 45 (10.7%). Of total study participants, about 205 (48.9%) had history of used RH service. More than half of those polled (273, or 65.2%) were third-year students, while 59, or 14.1%, were first-year students. About 206 (49.2%) of participants lived with their father and mother, but 138 (32.9%) had never discussed sexual and reproductive health, and 321 (76.6%) had enough pocket money to pay for the privilege. The majority of respondents (48.5%) were from a business college (Table 1).

RETRACTED

**Table 1:** Socio-demographic characteristics of undergraduate students of Addis Ababa University Addis Ababa, Ethiopia 2022

Variables	Frequency	Percept
Sex		
Male	198	47.3
Female	221	52.7
Age		
Less than or equal 18	3	0.7
19–24	371	88.5
Greater than 24	45	10.7
Academic years		
1st year	59	14.1
2nd year	87	20.8
3rd year	113	27
4th year	72	17.2
5th year	88	21
School of study		
College of law	97	23.2
College of business	203	48.4
College of COTTUM	119	28.4
To whom live		
With father and mother	206	49.2
With my mother only	32	7.6
With my father only	18	4.3
With relatives	29	6.9
With friends (dormitory)	79	18.9
Alone	55	13.1
Frequency of discuss to sex		
often	86	20.5
Occasionally	193	46.1
Never	138	32.9
Others specify	2	0.5
Pocket money		
Yes	321	76.6
No	98	23.4

### Knowledge and practice of RH service

Utilization of SRH services this study result showed that 205 (48.9%) of overall study subjects had received at least one component of the SRH services in the studied period. Majority of the participants 98 (23.4%) reported privet health facilities from where they received SRH services followed by governmental health facilities 80 (19.1%). The most frequently utilized SRH services were Volunteer Test and Counselling 80 (19.1%) and condom use 99 (23.6%). Table 2 shows in details.

**Table 2:** utilization of SRHS undergraduate students of Addis Ababa University, Ethiopia 2021

Variables	Frequency	Percent
What service did you used		
Family planning	60	14.3
*STD treatment*	38	9.1
VCT for HIV/AIDS	80	19.1
Abortion service	27	6.4
Post-abortion services	7	1.7
ANC	5	1.2
Condom use	99	23.6
Not ever utilized SRHS	192	45.8
Convenient time for SRHS		
As usual health institute working	245	58.5
In the hours when other users are not around	145	34.6
Other specify	29	6.9
What do you prefer on service fees for youth		
At usual rate	61	14.6
With discount for youth	104	24.8
Free of charge	243	58
Other specify	11	2.6
Whom be youth RH provider		
Young provider of the same sex	153	36.5
Young provider of any sex	87	20.8
Adult provider of the same sex	66	15.8
Any provider could be	103	24.6
Other specify	10	2.3
Prefer place for youth RH		
Anywhere out of resident area	224	53.5
In the centre of the town	92	22
At the school campus	96	22.9
Other specify	7	1.6
Where RH service get		
Government health centre	80	19.1
Private health facilities Family guidance association	98	23.4
School (campus) students clinic	22	5.6
Private health facilities	65	15.5

After a serious of questions regarding SRHS and reason why they not want to used SRHS respondents were asked whether they have had utilized SRHS in their life time see detail in Fig. 1

RETRACTED

**Fig. 1:** Reasons not to utilize SRHS by undergraduate students of Addis Ababa University, Ethiopia: 2022

As Fig. 2 revealed that 205 (48.9%) respondents were utilized SRHS in their life.

**Fig. 2:** History of SRHS utilization in their life among undergraduate students of Addis Ababa University, Ethiopia: 2022

A composite score including the 23 questions was developed to reflect the overall knowledge of the respondents. The finding indicates that 166 (39.5%) of the respondents could only answer up to 50 percent of the questions correctly. With regard to attitude, of the total 7 composite attitude scores, the mean attitude score was found to be more than 3 out of 7. The large majority (257, or 61.3%) could only answer correctly.

Only 206 (49.2%) of the total 419 participants have knowledge of SRH services.174 (41.5%) of participants used family planning methods; 37.5% used either abortion or post-abortion services; but about 3.3% do not know which PRH services were utilized.

The overall knowledge status regarding sexual reproductive health service utilization among study participants was 39.6%, with a 95% CI ranging from 34.4 to 44.6% (see details in Fig. 3).

**Fig. 3:** Knowledge status of undergraduate students of Addis Ababa University toward sexual Reproductive health service utilization, Ethiopia 2022

Participants were asked important questions about the reasons, timing, judgment, and confidentiality of RH services in order to assess their attitude toward RH service utilization. Finally, 257 (61.3%) of respondents had a favorable attitude toward the SRH services. The overall positive attitude status toward sexual and reproductive health service utilization among study participants was 61.3%, with a 95% CI of 41.9–92.4%; see Fig. 4 for details.

**Fig. 4:** Attitude status of undergraduate students of Addis Ababa University toward sexual Reproductive health service utilization, Ethiopia 2022

### Factors associated with utilization of RH service

The variables are attitude, knowledge, and satisfaction; college of education; who lives; discussion; and location; and which wards SRHS were significant in binary analysis, as indicated by p values less than 0.05 in the table below, and were entered into multivariable logistic regression to minimize the effect of confounders. Independent predictors of SRH service were identified, as shown in Table 3. In comparison to those in colleges of business, they used SRHS nearly 3.55 times less than those in colleges of law (AOR (95% CI) 3.546 (1.62–7.79).

RETRACTED

**Table 3:** Factors associated with utilization of RH service among undergraduate students of Addis Ababa University, Ethiopia: 2022

Variables	RH utilization		AOR (95% CI)	*P* value
	Yes	No		
College/school of study				
Low college	57 (13.6)	40 (9.5)	1	
Business college	117 (27.9	86 (20.5)	3.55 (1.62–7.79)	0.002
COTTUM college	83 (19.8)	36 (8.6)	1.81 (0.886–3.708	0.104
Frequency of discuss to sexual reproductive health-related issues with your family, friend				
Often	49 (11.7)	37 (8.80)	1.93 (3.346–1.12)	0.017
Occasionally	100 (23.8)	93 (22.2)	1.232 (2.05–0.73)	0.425
Never	56 (13.30)	84 (20)	1	
Convenient location of Youth RHs				
Yes	203 (48.45)	2 (0.48)	8.31 (1.61–42.93)	0.011
No	201 (47.97)	13 (3.1)	1:00	
Fee of RH services				
No	119 (28.4)	86 (20.52)	12.34 (6.48–23.49)	0.000
Yes	31 (7.4)	183 (43.68)	1:00	
Satisfied to received RH services				
No	161 (38.42)	42 (10.02)	1	
Yes	87 (20.76)	122 (29.12)	4.59 (2.54–8.33)	0.000
Knowledge				
Poor	116 (27.6)	89 (21.2)	1	
Good	50 (11.9)	164 (39.1)	4.17 (2.27–7.64)	0.000
Attitude				
Negative	91 (21.7)	114 (27.2)	1	
Positive	71 (16.9)	143 (34.1)	3.15 (1.71–5.8)	0.000
To whom live				
With father and mother	86 (20.52)	120 (28.6)	1	
With mother	23 (5.49)	9 (2.15)	9.4 (2.78–31.5)	0.000
With father	10 (2.39)	8 (1.91)	1. 12 (0.31–4.54)	0.805
With relative	17 (4.06)	12 (2.86)	2.74 (0.97–27.77)	0.058
With friend	29 (6.92)	50 (11.93)	0.84 (0.41–1.75)	0.650
Alone	40 (9.55)	15 (3.58)	5.75 (2.40–13.79)	0.000

Respondents who live with only their mother used the SRHS 9 times more than those who live with both their father and mother (AOR (95% CI) 9.37 (2.78–31.51) and 5.75 (2.40–13.79), respectively).

Simultaneously, respondents with a positive attitude toward the SRHS are three times more likely to use it than the counter AOR (95% CI) of 3.15 (1.71–5.80).

Knowledge was another important factor: respondents with good knowledge were used four times more than the counter (AOR (95% CI) 4.16 (2.27–764).

## Discussion

Adolescence is a developmental period marked by sexual discovery and often by sexual risks. A principal means for transmitting sexual values, beliefs, expectations, and knowledge between parents and their adolescents is through discussion. The relevance of SRHS for youth is emphasized in different studies. In countries in various regions of the world and with different development levels, this institution-based cross-sectional study tried to assess SRH utilization and identify factors associated with utilization of adolescent reproductive health services, including socio-demographic, knowledge, attitude, and institution-based factors, as well as adolescents’ awareness about the services in Addis Ababa University, Ethiopia. There is a lower rate of SRHS utilization among young and adolescent women, the period of life in which they are most sexually active, most fertile, and thus most exposed to sexual risk. However, having these risks makes the majority of them vulnerable to having their lives disrupted due to a variety of factors. This study determined the prevalence of utilization of sexual reproductive health services was low with identified factors increases attitude, knowledge, satisfaction, discussion and location toward SRHS likelihood utilization of sexual reproductive health services. In this study among 419 respondents, about 205 (48.9%) have had one or more time utilized SRHS in their life. This finding was higher than over all SRHS user in Study done in Bahir Dar city Ethiopia, 32% [14], Nekemte town, East Wallaga, Ethiopia (21.2%) [15] and Harar Town, in Ethiopia (63.8%) [16].

RETRACTED

The possible reason for the discrepancy might be due to respondent characteristics, socio-demographic backgrounds, and the time reference used in the definition of SRH service utilization. A high SRHS utilization rate in Addis Abeba might be the result of the availability of a larger number of private health centers, social doctors, and drug vendors. In addition, the fact that sex-related issues are stigmatized in Ethiopian society, especially in rural areas, means that a lot of underreporting can be expected, particularly in home-based surveys when questions require individuals to report on SRHS utilization, which is usually done by resident enumerators in national surveys. Other reasons for this could be due to study design, sample size, and methodology differences. Differences in the availability of services, the level of stigma surrounding them in society, the degree of women's access to information, and women's socioeconomic status were also related to the social and legal context of SRHS. This study’s findings, the result is lower than studies done in Mandalay City, Myanmar (67%) [17], West Arsi Zone in Oromia region, Ethiopia (58.6%) [18], study in Addis Ababa, Ethiopia, (67.8%) [19] had ever utilized at least one type of RH service. The disparity could be attributed to the small number of facilities and the need to discover more. This could also be due to differences in study design and methodology.

In this study, nearly 3.55 times as many respondents used SRHS as those in college of law (AOR (95% CI) 3.546 (1.62–7.79) compared to those in college of business). This could be due to the fact that most students from businesses may have more knowledge or awareness about sexual and reproductive health services. Besides, the students may also perceive the long queue, location, and dissatisfaction as normal, and additional studies using qualitative designs may be needed to dig out the deeper meaning and identify the type of information delivered by the college. This finding is consistent with evidence from studies conducted in different parts of Ethiopia [11, 20] and Ghana [21]. This study result shows that those who were not living with the family used SRH services more frequently. Respondents who live with only their mother used the SRHS 9 times more frequently than those who live with their families (AOR (95% CI) 9.37 (2.78–31.51) and 5.75 (2.40–13.79), respectively). This explains that living with family and being under parental control may protect students from early sexual exposure and unwanted sexual activity, and they may also be more likely to find themselves with a peer who would perpetuate such an act in separated parenthood for those who live without family. Findings were consistent within Nekemte Town, Ethiopia [22] and Kenya [23]. Simultaneously, respondents with a positive attitude toward the SRHS are three times more likely to use it than the counter AOR (95% CI) of 3.15 (1.71–5.80). Another important factor was knowledge; as shown in Table 3, the respondent with good knowledge was four times more utilized than the counter (AOR (95% CI) 4.16 (2.27–7.64). Lack of knowledge and a negative attitude toward SRHS are some of the possible barriers to low utilization of SRHS. Young people know very little about reproductive health and their own biology and are often victims of their own misconceptions about the risks and dangers of unsafe sexual relations [17]. Only 13.9% of rural study subjects and 24.5% of urban study subjects correctly identified a woman as most likely to become pregnant halfway between two periods, which is lower than Harar and Addis Abeba findings [5, 24]. In this study, we found that family factors, as well as individual and reproductive factors, played an important role in youths’ utilization of RH services. Youths who frequently discussed AOR with friends and family members were nearly twice as likely to use SR services as those who never discussed AOR (95% CI 1.93; 3.346; 1.12); this can be justified by the fact that discussion of services with family and friends allows youths to create more opportunities to exchange information, share experiences, and build comprehensive knowledge about SRHS. It can also create opportunities to deal with adolescent problems associated with SRH service utilization so that health professionals might be the source of accurate information for youths, which helps them make appropriate decisions about their seeking behavior for health services. This finding was supported by one study that found that the relationship between youths and their parents, as well as childhood family conditions, influenced the youth’s utilization of RH services in different areas [21, 24]. Respondents who were able to easily obtain convenient locations for SRHS used them more than eight times more than counters in AOR (95% CI 8.31; 1.61–42.93), and it can be predicted that as youths become more familiar with the service settings as well as the types of services offered, they freely decide what type of service they have to use and why, when, and where to use [5, 11], whereas financial deprivation hampered SRHS utilization among users, and these findings indicate that inaccessibility to SRH services due to location and financial aspects has been present in the study area [8]. In this study, satisfaction with SRH services was found to be more important than location and payment. It was found that those respondents who had satisfaction greater than 4 were more likely to utilize reproductive health services than those who had satisfaction AOR (95% CI 4.59; 2.54–8.33), and this finding was supported by a study done at [11]. This might be because those who ever had satisfaction might need further relevant services to avoid the risk and consequences of sexual vulnerability. This study was also susceptible to recall bias, as its participants may not have been able to accurately remember issues from the past. This cross-sectional study cannot explore the temporal relationship.

RETRACTED

## Conclusion

This study discovered that the prevalence of sexual reproductive health service utilization was low, with identified factors increasing SRHS likelihood utilization of sexual reproductive health services by increasing attitude, knowledge, satisfaction, discussion, and location. Poor knowledge and a negative attitude toward SRHS were threats of harm that contributed to the health problems that adolescents face nowadays, including abortion, STDs, and unwanted pregnancies. This study also discovered that the main reasons for these populations not using sexual reproductive health services were location, time, and cost. An increased effort was required to improve adolescent reproductive health utilization. Therefore, policymakers and health planners would be better off strengthening the urgent need to ensure adequate SRHS through knowledge and attitude building. This represents a greater burden in terms of preventing and managing this health issue.

RETRACTED

Policymakers and health planners should work to integrate reproductive health education at the primary, secondary, and university levels. Policymakers should emphasize the need for adequate SRHS, knowledge, and attitude building among Ethiopian undergraduate students in higher education, as well as serve as advocates for SRHS services and make them available at a nearby location. Health planners should also raise awareness among adolescents that sexual risk is a serious problem that can harm their future lives. Addis Ababa University should work on establishing and strengthening adolescent reproductive health clubs on and off campus, and student health centers should provide sexuality education, family planning, and reproductive health services to increase SRHS utilization.

## Data Availability

Datasets used in the current study are available from the corresponding author upon reasonable request.

## Abbreviations

AOR: Adjusted odd ratio
CI: Confidence interval
EDHS: Ethiopian Demographic and Health Survey
FMOH: Federal ministry of health
HIV: Human Immune-Deficiency Virus
IEC: Information Education and Communication
NGO: Non-Governmental Organization
OR: Odds ratio
RH: Reproductive health
SRHS: Sexual and reproductive health service
STI: Sexually transmitted infection
VCT: Voluntary counselling and testing
WHO: World Health Organization
